# Effects of Tenofovir Combined with Recombinant Human Interferon *α*-2b on Negative Conversion Rate, Liver Function, Immune Status, and Drug Safety in Patients with Chronic Hepatitis B: A Systematic Review and Meta-Analysis

**DOI:** 10.1155/2022/1889628

**Published:** 2022-06-30

**Authors:** Hui Zhang, Jianchun Xian, Yang Li, Li Xiao, Lu Wang

**Affiliations:** ^1^The Medical Department of Hepatology, Jiangsu Taizhou People's Hospital, Taizhou 225300, China; ^2^The Medical Department of Neurology, Jiangsu Taizhou People's Hospital, Taizhou 225300, China

## Abstract

**Objective:**

To systematically evaluate the clinical value of tenofovir combined with recombinant human interferon *α*-2b in the treatment of chronic hepatitis B and to provide evidence-based medicine for its popularization and use.

**Methods:**

The randomized controlled trials (RCTs) of tenofovir combined with recombinant human interferon *α*-2b in the online database of PubMed, EMBASE, ScienceDirect, Cochrane Library, China knowledge Network (CNKI), China VIP database, Wanfang database, and China Biomedical Literature Database (CBM) were searched. The data included in this study were extracted by two independent researchers. After extracting the data of the study, the Cochrane manual 5.1.0 standard was used to evaluate the bias risk of all the literature included in this study. RevMan5.4 statistical software was used to analyze the collected data by meta.

**Results:**

Entecavir combined with recombinant human interferon *α*-2b can inhibit the activity of HBV polymerase and improve the inflammatory response of the liver. Recombinant human interferon *α*-2b can regulate immune function by inducing T cell differentiation and maturation and enhancing the production of cytokines. The systematic evaluation showed that entecavir combined with recombinant human interferon *α*-2b had higher serum HBeAg negative conversion rate, higher drug safety compared with entecavir alone, and improved liver function and immune status.

**Conclusion:**

Tenofovir combined with recombinant human interferon alpha-2b has a high serum HBeAg negative rate and safety profile for the treatment of chronic hepatitis B. The combination treatment can improve liver function and immune status in patients, but more studies with higher methodological quality and longer duration of intervention are needed for further validation.

## 1. Introduction

Chronic hepatitis B (CHB) is a viral infectious disease that seriously endangers human health [1]. According to the statistics of the World Health Organization (WHO), there are about 350 million people with chronic HBV infection in the world [2, 3]. About 80% of the patients have varying degrees of hepatocyte damage and may develop cirrhosis and liver cancer [4]. WHO has listed HBV infection as one of the top 10 contributors to death in the world [5]. The number of people dying from chronic hepatitis B (or secondary liver cirrhosis or hepatocellular carcinoma) reaches 500000 to 1.2 million every year [6]. China is a high prevalence area of HBV and the positive rate of HBsAg in the general population is 9.09% [7]. Additionally, the positive rate of HBsAg in people vaccinated with and without the hepatitis B vaccine is 4.51% and 9.51%, respectively, and most of them are perinatal infections (through mother-to-child transmission). HBV is very harmful because it can constantly replicate itself, which allows it to persist, and these factors can lead to the progression of HBV disease. Studies have found that patients who are infected with HBV before the age of 6 are more likely to develop cirrhosis in adulthood, which is known to eventually lead to liver cancer. Based on the above reasons, the focus of the treatment of chronic hepatitis B is anti-HBV.

HBV belongs to hepatoviridae and has a circular partial double-stranded DNA with a molecular weight of 3.2 kb. The DNA molecule contains four open reading frames (ORF) that encode capsid protein, membrane protein, polymerase, and X protein, respectively. Hepatitis B virus particles are composed of hepatitis B virus nucleic acid and outer membrane. In the process of hepatitis B virus replication cycle, hepatitis B virus particles firstly bind to the receptor hydroxypeptidase D on the cellular membrane and enter the cell. Then, the capsid is removed by phosphorylation of the capsid protein. In the end, the hepatitis B virus enters the nucleus and is transformed into superhelix DNA (cccDNA) in the nucleus. Covalently closed circular DNA (cccDNA) is the template of hepatitis B virus transcription, which can transcribe mRNA. The previous gene RNA is used as a template and the negative strand of hepatitis B virus DNA is synthesized by reverse transcription outside the nucleus and then the positive strand of hepatitis B virus DNA is synthesized. The hepatitis B virus in the capsid is encapsulated by the membrane and secreted outside the cell to enter other human cells with complete virus particles. It can also be re-stripped off the capsid into the human nucleus to maintain the number of cccDNA in the nucleus. After HBV infection, the immune response determines the occurrence, development, and prognosis of hepatitis B. HBV can be replicated continuously in the human body, resulting in chronic immune tolerance, so the virus is not easy to be eliminated [8].

Currently, it is recognized that the complete or incomplete immune tolerance of the host to various antigens of HBV is the main reason for the chronicity of HBV infection [9]. Under normal circumstances, Th1/Th2 is in dynamic equilibrium and the imbalance of the Th1/Th2 ratio is one of the main factors governing the effectiveness of the body in eliminating viruses and virus-infected cells [10]. During chronic HBV infection, disruption of Th1/Th2 cytokines, especially defective production of Th1 cytokines such as IFN-a, IL-2, and IL-12, leads to a decrease in cellular immune function and helper B-cell function during HBV infection, making it difficult to clear the virus. If the Th1 cell subpopulation is dominant, it will promote a cellular immune response, enhance the activity of CD+ cells, and clear intracellular viruses, but it will also exacerbate hepatocyte damage and cause acute or self-limiting inflammation. If Th2 cells are dominant, it will promote humoral immune response and inhibit the cellular immune response to weaken the activity of CTL cells resulting in persistent inflammation. HBV infection does not induce a single change of Th1 or Th2, but an imbalance of Th1/Th2. Therefore, to adjust the balance of Th1/Th2 and to enhance the level of Th1 cells is also one of the key points in the treatment of hepatitis B. Currently, the overall goal of international antiviral treatment for chronic hepatitis B is to maximize long-term suppression or elimination of HBV, delay disease progression and prevent the development of cirrhosis, HCC, and their complications, thereby prolonging survival and improving quality of life [11–13]. Therefore, the measures to treat hepatitis B virus infection include antiviral therapy, which is considered to be the current strategy of choice. The main antiviral drugs are nucleotide antivirals (NUC) or interferon (IFN-*α*) [14]. The advantages of interferon therapy are a fixed course of treatment, a relatively high rate of antigen conversion, and a relatively low incidence of rebound after discontinuation; the disadvantages are widespread drug resistance and significant adverse effects. The advantages of NUCs treatment are ease of administration, few adverse effects, and good tolerability; the disadvantages are the relatively long duration of treatment, common drug resistance, and high relapse rate after discontinuation of the drug. Among them, entecavir (ETV) in NUCs has been replaced by telbivudine, adefovir, and lamivudine as the first-line oral drugs for patients. The reverse transcription controls HBV replication and slows the risk of HCC progression and HBV-related death. However, HBV cannot be completely cured, because HBV cccDNA cannot be completely eliminated [15]. In addition to the above, the study also found that long-term treatment of NUC is currently the routine treatment for patients with HBV. After the emergence of ETV, it has become a clinical first-line antiviral drug, the drug that has a good effect on the treatment of hepatitis B virus. Inhibition or blockade of hepatitis B virus replication and transcription is also a therapeutic strategy, such as inhibition of hepatitis B virus nucleoside polymerase activity. On this basis, our study provides more reliable evidence-based clinical evidence through a meta-analysis of the effects of tenofovir, combined with recombinant human interferon alpha-2b, on negative regression rates, liver function, immune status, and medication safety in patients with chronic hepatitis B.

## 2. Research Contents and Methods

### 2.1. Sources and Retrieval Methods of Documents

From the establishment of the database to the present, the Chinese Journal full-text Database (CNKI), VIP full-text Database (VIP), Wanfang Database, and Chinese Biomedical Literature data (CBM) were searched. The relevant Chinese journals, conference papers, and degree papers were searched. The data of tenofovir combined with recombinant human interferon *α*-2b in the treatment of chronic hepatitis B in China were collected. Literature retrieval was conducted in the form of free words + subject words with the keywords of tenofovir, recombinant human interferon *α*-2b, chronic hepatitis B, and so on. The data included in this study were extracted by two independent researchers. After extracting the data of the study, the Cochrane manual 5.1.0 standard was used to evaluate the bias risk of all the literature included in this study.

### 2.2. Inclusion and Exclusion Criteria of Literature

#### 2.2.1. Literature Inclusion Criteria

1. Study type was all domestic randomized controlled trials (RCT) of tenofovir combined with recombinant human interferon *α*-2b in the treatment of chronic hepatitis B and entecavir. The language was limited to Chinese.
2. Subjects: HBeAg positive patients met the diagnostic criteria of chronic hepatitis B in the guidelines for prevention and treatment of chronic hepatitis B [16].
3. Intervention: the observation group was treated with tenofovir combined with recombinant human interferon *α*-2b and the control group was treated with tenofovir.

#### 2.2.2. Document Exclusion Criteria

1. It was not a randomized controlled study.
2. The data report was incomplete and the data could not be used.
3. Repeated the research content and the latest research.
4. The evaluation of the curative effect of the study was not significant.

### 2.3. Quality Evaluation and Data Extraction

1. Bias risk assessment included in the study. The bias risk assessment tool recommended by Cochrane system Review Manual 5.3 was used for evaluation.
2. Literature screening and data extraction. Two researchers independently screened the literature, extracted the data, evaluated the quality, and cross-checked. In case of differences, they discussed and resolved or asked the third researcher to assist in judgment. Note: express document management software and Excel office software were used to manage and extract research data if the data included in the literature was incomplete. The author of this article would be contacted to supplement it. The content of data extraction included (1) basic information: author(s), publication time, and the number of cases; (2) intervention measures: dose and course of treatment; (3) outcome index.

### 2.4. Statistical Processing

RevMan5.3 software was used for meta-analysis. Relative risk (OR) was used as the effective index for counting data and mean difference (MD) was used as the effective index for measuring data. The point estimate and 95% confidence interval (CI) of each effect were given. *χ*^2^ test was used for the heterogeneity test and I2 was used to judge the heterogeneity. If there was no heterogeneity, the fixed-effect model was used; if there was heterogeneity, subgroup analysis, sensitivity analysis, or descriptive analysis was used, and the random effect model was used. *P* < 0.05 indicates that the difference was statistically significant.

## 3. Results and Analysis

### 3.1. The Results of Literature Retrieval and the Basic Situation of Literature Inclusion

A total of 451 articles were retrieved through a computer database, of which 175 articles were obtained after eliminating repeated studies and 89 articles were obtained from a preliminary reading of titles and abstracts, and 33 articles were included after excluding irrelevant studies, reviews, case reports, and non-control articles. In addition, 26 articles with incomplete data and no main outcome indicators were read carefully and finally included 7 RCT [17–23]. A total of 750 samples were analyzed by meta.

### 3.2. Evaluation of the Quality of Methodology Included in the Literature

Of seven RCT literature in this meta-analysis that reported the baseline status of patients, only two RCT studies mentioned random assignment. However, the random method did not explain anything and the rest did not mention “random” information. The five studies that were included gave detailed intervention measures and follow-up time. The number and reasons for the blind method and loss of follow-up or withdrawal were not described in detail in seven RCT articles. According to the Jadad scale, it was found that all the seven articles had RCT ≤2points.

### 3.3. Results of Meta-Analysis

#### 3.3.1. HBeAg Negative Conversion Rate

Through the inclusion of 7 RCT studies, the lower limb scores of Fugl–Meyer motor function evaluation between the experimental group and the control group were analyzed by meta-analysis. The results of the heterogeneity test showed that Chi^2^ = 4.34, df = 4, *P*=0.31 > 0.05, *I*^2^ = 16%, indicating that there was no obvious heterogeneity among the included research data. The combined effect of WMD was analyzed by a fixed-effect model. The combined effect of WMD was 5.96 and the confidence interval of 95% was (5.77, 6.15, Figure 1), and the test of combined effect dose WMD was *Z* = 62.24 (*P* < 0.00001). According to the results of this analysis, it can be considered that there is a significant difference in the WMD of tenofovir combined with recombinant human interferon *α*-2b compared with tenofovir in the treatment of patients with chronic hepatitis B and the 95% confidence line of WMD fell on the right side of the invalid line, indicating that the negative conversion rate of tenofovir combined with recombinant human interferon *α*-2b was higher than that of tenofovir in patients with chronic hepatitis B.

#### 3.3.2. Drug Safety

The drug safety scores between the experimental group and the control group were analyzed by meta. The results of the heterogeneity test showed that Chi^2^ = 4.34, df = 4, *P*=0.31 > 0.05, *I*^2^ = 16%, indicating that there was no heterogeneity among the included research data. In addition, the combined effect of WMD was analyzed by the fixed-effect model. According to Figure 2, the combined effect of WMD was 2.66 and the confidence interval of 95% was (2.60, 2.72), and the test of the combined effect dose WMD was *Z* = 82.12 (*P* > 0.05). According to the results, it can be considered that there was no difference in the safety of tenofovir combined with recombinant human interferon *α*-2b and tenofovir in the treatment of patients with chronic hepatitis B.

#### 3.3.3. Liver Function

The effects of liver function between the experimental and the control groups were analyzed by meta. The heterogeneity test showed that Chi^2^ = 4.34, df = 4, *P*=0.31 > 0.05, *I*^2^ = 16%, indicating that there was obvious heterogeneity among the included research data. The combined effect of WMD was analyzed by a random effect model. According to Figure 3, the combined effect of WMD was 1.06 and the 95% confidence interval was (0.94, 1.18). And the WMD test of combined effect was *Z* = 17.52 (*P* > 0.05). There was no difference in the effect of tenofovir combined with recombinant human interferon *α*-2b and tenofovir on liver function in patients with chronic hepatitis B. In this study, because there are few literature in line with the research conditions, and finally included in the analysis of the literature, so it does not meet the conditions for the funnel chart.

## 4. Discussion

Hepatitis B virus (HBV) is a common clinical disease. With the increase in its incidence, it has become a serious disease threatening human health. The global HBV infection rate (susceptibility to infection + previous infection) has reached 33% among more than 6 billion people worldwide. At least 2 billion people are infected with or have been infected with HBV, of which about 350 million chronic HBV infections are mainly distributed in Latin America, Africa, and Asia. Up to one million people worldwide die of liver cirrhosis or liver cancer caused by HBV infection every year [24, 25]. An epidemiological survey of HBV was conducted in China in 2006. The results showed that the carrying rate of HBsAg among people aged 1 to 59 years old was 7.18%. Since the 1990s, China has started to implement the HBV vaccination program, which has greatly reduced the number of people infected with HBV in our country. China has implemented this plan, and the transmission status of hepatitis B virus in China has been downgraded to a moderate level. At present, according to research reports, there are about 93 million people with HBV infection in China, of which 20 million are patients with chronic hepatitis B (CHB), accounting for the main part of HBV infection [26]. According to statistics, there are about 500000 to 1 million new cases of HBV infection in China every year, and the annual death toll is about 300000. The main routes of transmission of HBV include mother-to-child transmission, blood/humoral transmission, and sexual contact transmission. Mother-to-child transmission includes intrauterine infection, perinatal transmission, and postpartum transmission. In addition, a few studies have confirmed that HBV can be transmitted by blood-sucking insects such as mosquitoes. For HBV patients, history of blood transfusion, history of contact with HBV infection, history of dirty injections, and family history of the disease (especially mother's history of HBV carrier) are more helpful for clinical diagnosis. At present, acute hepatitis B is relatively rare. If HBsAg is positive for more than 6 months, the previous history of HBV infection, and current HBV/HBsAg diagnosis is positive, chronic hepatitis B infection can be diagnosed. The classification method is as follows [27]: (1) chronic hepatitis B is divided into HBeAg positive chronic hepatitis B and HBeAg negative chronic hepatitis B; HBeAg positive chronic hepatitis B:ALT (glutamic pyruvic transaminase) of the patients shows repeated or continuous increase, serum HBVDNA, HBsAg and HBeAg are positive, HBeAb test is negative, and liver biopsy shows inflammatory activity. HBeAg negative chronic hepatitis B:ALT shows a recurrent or persistent abnormality, serum HBVDNA and HBsAg are positive, HBeAg test is persistent negative, and liver biopsy shows inflammatory activity. According to the clinical manifestations and examination, chronic hepatitis B can be further divided into severe, moderate, and mild [28]. In addition, there are repeated inflammatory activities in the liver of patients with chronic hepatitis B, which will lead to large area necrosis of liver cells and proliferation of connective tissue in the liver and then lead to the emergence of liver cirrhosis and hepatitis. With the progress of the disease, liver cirrhosis can develop into decompensation, which leads to gastrointestinal bleeding and other symptoms, seriously affecting the quality of life. (2) The HBsAg test is negative in patients with occult chronic hepatitis B, but the liver/serum contains hepatitis B virus, and the clinical manifestations are the same as those in patients with CHB, such as nausea, fatigue, and loss of appetite. It may be accompanied by positive HBeAb and/or HBcAb and HBsAb tests. In addition, about 20% of occult CHB patients show negative serum markers, and only hepatitis B virus test is positive [29]. (3) HBV carriers: serum HBVDNA and HBsAg of chronic HBV carriers are positive and HBeAg/HBeAb are positive. These patients are immune tolerance carriers if the levels of ALT and AST are normal for three consecutive times within a year. And there is no obvious inflammatory activity in the liver, it is likely to be the immune tolerance stage. The features of inactive HBsAg carriers include HBsAg test being positive, HBeAg test being positive, and HBVDNA level being lower than the lowest range or cannot be detected because the content is too low. ALT levels are normal for three consecutive times within a year and there is a mild inflammatory activity in the liver.

For CHB patients, a positive HBeAg test indicates that they are in an active disease state according to a number of studies [30]. For CHB patients, the probability of disease progression to liver cancer and liver cirrhosis in HBeAg positive patients is higher than that in HBeAg negative patients. Therefore, antiviral therapy for diagnosed CHB patients should be carried out as soon as possible to effectively inhibit the replication process of HBVDNA [31]. For CHB patients, if the virus replication activity of HBeAg positive patients is higher than that of HBeAg negative patients, they have a higher HBVDNA load and liver cells are damaged more seriously, and the ability of virus transmission is higher, so active antiviral therapy should be carried out for these patients. For the treatment of HBeAg positive CHB patients, serological conversion of HBeAg negative is the most important treatment goal. In addition, it should be guaranteed to reduce the level of HBVDNA, promote the recovery of liver function, and ensure that the disease tends to be stable. At present, the clinical drugs used for anti-HBV are interferons, nucleoside (acid) analogues, and immunomodulators. Nucleoside (acid) analogues are represented by lamivudine (Lamivudine, 3TC), including entecavir (ETV), adefovir (ADV), and so on. These drugs have ideal antiviral strength and do not have serious and obvious side effects. They exert an anti-HBV effect by inhibiting the activity of HBVDNA reverse transcriptase and DNA polymerase [32]. It has been found that hepatitis virus in patients with chronic hepatitis B can be integrated into the nucleic acid of hepatocytes through transcriptional behavior and form a new HBVDNA by RNA reverse transcription. This kind of viral DNA cannot work completely by antiviral drugs alone. In addition to the above phenomena, a large number of long-term clinical use of NAs drugs will cause viral drug resistance, which will lead to poor clinical efficacy in the treatment of chronic hepatitis B. Taking the use of LAM as an example, it has been reported in the literature after 4 years of continuous treatment with LAM, the drug resistance rate was as high as 66% [33]. Marcellin et al. studied the effect of ETV on chronic hepatitis B patients and found that for patients receiving the drug for 7 years, regardless of whether the initial HBeAg test was negative or positive, the drug resistance rate was 0%, and 99% of patients had HBVDNA <400 copies/ml [40]. Furthermore, for HBeAg positive CHB patients, the serological response rate increased with the increase of ETV medication time and the serum HBeAg conversion rate was more than 40% in patients who had been using ETV for 7 years. Marcellin et al. studied the liver histology of HBeAg positive CHB patients who received continuous ETV treatment for 5 years [34]. Liver biopsies were performed in 384 newly treated CHB patients before and 5 years after treatment. The results showed that 96 patients were cirrhotic before treatment and 252 patients did not develop liver cirrhosis. Five years later, 71 patients reversed cirrhosis with a reversal rate of 74%. A total of 239 patients achieved the prevention of the progression of liver fibrosis with a tissue rate of 95%. Therefore, it has been pointed out that for HBeAg positive CHB patients, long-term use of ETV can prevent liver fibrosis and reverse liver cirrhosis [35]. Interferon (IFN) is a trace protein with high biological activity, which is generally divided into type I, type II, and type III [33]. Interferon is a kind of broad-spectrum antiviral drug, which does not directly kill or inhibit the virus in practical use. Interferon can make cells produce antiviral proteins through the action of cell surface receptors, thus inhibiting virus replication. At present, the common clinical types of interferon are a (leukocyte) type, *β* (fibroblast) type, and *β* (lymphocyte) type. Type I interferon mainly includes IFN-*α*, IFN-*β*, IFN-*ω*, and so on. IFN-*α* is a polypeptide with a relative molecular weight (MW) of 18000 produced by monocytes. It can neutralize viruses or eliminate virus-infected cells by inducing an antiviral state and regulating the immune system in cells. According to the different amino acid sequences, IFN-*α* can be divided into IFN-*α*-1b, IFN-*α*-2a, and IFN-*α*-2b. In clinical therapy, interferon enhances the viability of natural killer cells, T-lymphocytes, and macrophages, thus acting as an immunomodulatory agent. Therefore, the use of interferon can have a strong anti-hepatitis B virus effect on patients with hepatitis B cirrhosis, to better improve the clinical symptoms of patients and the development of liver cirrhosis, which is of great significance [36]. In particular, the 2015 APASL guidelines recommend that interferon can be used for initial antiviral therapy in patients with pre-cirrhosis and interferon in compensatory cirrhosis [37]. The reasons are as follows: (1) interferon therapy can prevent the progression of liver cirrhosis; (2) interferon therapy can stop medication within a limited course of treatment; and (3) interferon therapy can improve the response rate of interferon. The ultimate goal is to delay the use of nucleoside drugs and variation of drug resistance, prolong the life of patients, and improve the quality of life through interferon therapy. However, it should be noted that the difference between pre-cirrhosis and typical cirrhosis and chronic hepatitis is very difficult. Misuse of interferon in patients with decompensated cirrhosis and middle and late-stage cirrhosis may induce chronic acute liver failure and threaten the safety of patients. Therefore, many doctors will not primarily choose it in clinical treatment but will only carry out routine treatment for patients. This may lead to the aggravation of the patient's condition and even further development of the patient's condition, which will pose a great threat to the patient's health and life [38].

A meta-analysis was conducted to explore the effects of tenofovir combined with recombinant human interferon *α*-2b on negative conversion rate, liver function, and drug safety in patients with chronic hepatitis B. A total of 7 RCTs were finally included and a total of 750 samples were analyzed by meta [17–23]. The results showed that entecavir combined with recombinant human interferon *α*-2b could inhibit the activity of HBV polymerase and improve the inflammatory response of the liver. Recombinant human interferon *α*-2b can regulate immune function by inducing T cell differentiation and maturation and enhancing the production of cytokines. The results of a systematic review of this study show that entecavir combined with recombinant human interferon *α*-2b has a better therapeutic effect. Compared with entecavir alone, this combination therapy can make patients' serum HBeAg negative conversion rate higher and safer during drug use. In addition, the synergistic effect of entecavir combined with interferon *α*-2b is better in improving liver function and immune status.

In conclusion, tenofovir combined with recombinant human interferon alpha-2b has a high serum HBeAg negative rate and safety profile for the treatment of chronic hepatitis B. The combination treatment can improve liver function and immune status in patients, but more studies with higher methodological quality and longer duration of intervention are needed for further validation [39].

## Figures and Tables

**Figure 1:** Forest plot of meta-analysis of the negative conversion rate of HBeAg.

**Figure 2:** Forest plot of meta-analysis of security.

**Figure 3:** Forest plot of meta-analysis of liver function score.

## Data Availability

No data were used to support this study

## References

[1] Wu Y., Cheng C., Lai W., Qiu Z., Zhang Li (2021). Effect of tenofovir combined with pegylated interferon *α*-2b injection on serological conversion rate and negative conversion rate of HBeAg in patients with chronic hepatitis B. *Advances in Modern Biomedicine*.

[2] Du J., Wang Y., Li win, Yang R., Zhao W. (2020). Effects of pegylated interferon *α*-2a combined with tenofovir axetil on collagen metabolism, YKL-40, MMP-2 and MMP-9 in patients with chronic hepatitis B. *Clinical Medical Research and practice*.

[3] Xiao F., Wang M., Zhou L., Yin F., Wang Z. (2020). Clinical observation of pegylated interferon *α*-2b combined with tenofovir in the treatment of HBeAg positive chronic hepatitis B for 48 weeks. *Journal of Aerospace Medicine*.

[4] Xu Y., Wu P. (2022). Efficacy and negative conversion rate of tenofovir combined with polyethylene glycol interferon *α* 2a in the treatment of chronic hepatitis B [J]. *Jilin Medicine*.

[5] Tang L. S. Y., Covert E., Wilson E., Kottilil S. (2018). Chronic hepatitis B infection:. *a review, JAMA, *.

[6] Xiao Li (2020). Effects of pegylated interferon *α*-2a combined with tenofovir axetil on the expression of serum Mig, RANTES and hepatic fibrosis markers in newly treated patients with high viral load of chronic hepatitis B [J]. *China Medical Herald*.

[7] Guo Z., he W., Pei J. (2019). Analysis of the efficacy of polyethylene glycol interferon *α*-2a injection combined with tenofovir axetil in the treatment of e-antigen positive chronic hepatitis B [J]. *Chinese Medicine and Clinic*.

[8] Duan H., Pu H., Yin G. (2020). Efficacy of tenofovir combined with pegylated interferon *α*-2 *α* in the treatment of ntecavir chronic hepatitis B [J]. *Gansu Medicine*.

[9] Zhao W., Yang R., Dou J., du J., Liu S., Li C. (2019). Efficacy of tenofovir axetil combined with polyethylene glycol interferon *α*-2b in the treatment of patients with chronic hepatitis B [J]. *Henan Medical Research*.

[10] Tang Y., Liang H., Zeng G. E., Shen S., Sun J. (2022). Advances in new antivirals for chronic hepatitis B. *Chinese Medical Journal*.

[11] Yang J. M., Chen L. P., Wang Y. J. (2020). Entecavir add-on Peg-interferon therapy plays a positive role in reversing hepatic fibrosis in treatment-naïve chronic hepatitis B patients: a prospective and randomized controlled trial. *Chinese Medical Journal*.

[12] Zhang H., Lu Y., Wu X. (2019). Effects of pegylated interferon *α* 2a combined with tenofovir on liver function and HBV-DNA negative conversion rate in patients with drug resistant hepatitis B [J]. *Chinese and Foreign Medicine*.

[13] Lan-Lan X., Wu X.-X., Jia-Jia C. (2021). Progress in hepatitis B virus-related acute-on-chronic liver failure treatment in China: a large, multicenter, retrospective cohort study using a propensity score matching analysis[J]. *International Journal of Hepatobiliary and Pancreatic Diseases*.

[14] Stornaiuolo G., Stanzione M., Brancaccio G. (2007). Viral blips during long-term treatment with standard or double dose lamivudine in HBe antigen negative chronic hepatitis B[J]. *World Journal of Gastroenterology*.

[15] Li M. H., Lu H. U., Chen Q. Q. (2021). Changes in the cytokine profiles of patients with chronic hepatitis B during antiviral therapy. *Biomedical and Environmental Sciences: Biomedical and Environmental Sciences*.

[16] Robaeys G., De Bie J., Wichers M. C. (2007). Early prediction of major depression in chronic hepatitis C patients during peg-interferon a-2b treatment by assessment of vegetative-depressive symptoms after four weeks[J]. *World Journal of Gastroenterology*.

[17] Xin J. I. N., Bin F. U., Wu Z. J. (2020). Serum chitinase-3-like protein 1 is a biomarker of liver fibrosis in patients with chronic hepatitis B in China[J]. *International Journal of Hepatobiliary and Pancreatic Diseases*.

[18] Yin X.-R., Liu Z.-H., Liu J. (2019). First line nucleos(t)ide analog monotherapy is more cost-effective than combination strategies in hepatitis B e antigen-positive chronic hepatitis B patients in China [J]. *Chinese Medical Journal*.

[19] Robaeys G., Bie J. D., Ranst M. V., Buntinx F. (2007). An extremely rare case of delusional parasitosis in a chronic hepatitis C patient during pegylated interferon alpha-2b and ribavirin treatment[J]. *World Journal of Gastroenterology*.

[20] Yao H. U., Ying-Zi Y. E., Ye L. J., Wang X. H., Yu H. (2019). Efficacy and safety of interferon alpha-2b versus pegylated interferon alpha-2a monotherapy in children with chronic hepatitis B: a real-life cohort study from Shanghai, China[J]. *World Journal of Pediatrics (English version)*.

[21] Li M. H., Zhang L., Qu X. J. (2017). The predictive value of baseline HBsAg level and early response for HBsAg loss in patients with HBeAg-positive chronic hepatitis B during pegylated interferon alpha-2a treatment[J]. *Biology and Environmental Science (English Version)*.

[22] Shi Y. H., Shi C. H. (2009). Molecular characteristics and stages of chronic hepatitis B virus infection[J]. *World Journal of Gastroenterology*.

[23] Matsumoto K., Miyake Y., Miyatake H. (2009). A combination treatment of entecavir and early-phase corticosteroid in severe exacerbation of chronic hepatitis B[J]. *World Journal of Gastroenterology*.

[24] You J., Sriplung H., Geater A. (2008). Effect of viral load on T-lymphocyte failure in patients with chronic hepatitis B[J]. *World Journal of Gastroenterology*.

[25] Li H., Wang H., Peng C. (2017). Predictors for efficacy of combination therapy with a nucleos(t)ide analogue and interferon for chronic hepatitis B[J]. *Journal of Huazhong University of Science and Technology (Medicine) (English-German version)*.

[26] Cai C. J., Chen H. A., Lu M. Q., Chen G. H. (2008). Model for end-stage liver disease-sodium predicts prognosis in patients with chronic severe hepatitis B[J]. *Chinese Medical Journal*.

[27] Lu G. F., Tang F. A., Zheng P. Y., Yang P. C., Qi Y. M. (2008). Entecavir up-regulates dendritic cell function in patients with chronic hepatitis B[J]. *World Journal of Gastroenterology*.

[28] Zhao Z. X., Cai Q. X., Peng X. M., Chong Y. T., Gao Z. L. (2008). Expression of SOCS-1 in the liver tissues of chronic hepatitis B and its clinical significance[J]. *World Journal of Gastroenterology*.

[29] Zhang Y. X., Wu W. J., Zhang Y. Z., Feng Y. L., Zhou X. X., Pan Q. (2008). Noninvasive assessment of liver fibrosis with combined serum aminotransferase/platelet ratio index and hyaluronic acid in patients with chronic hepatitis B[J]. *World Journal of Gastroenterology*.

[30] Nam S. W., Bae S. H., Lee S. W. (2008). Short-term overlap lamivudine treatment with adefovir dipivoxil in patients with lamivudine-resistant chronic hepatitis B[J]. *World Journal of Gastroenterology*.

[31] Papatheodoridis G. V., Manolakopoulos S., Archimandritis A. J. (2008). Current treatment indications and strategies in chronic hepatitis B virus infection[J]. *World Journal of Gastroenterology*.

[32] Lu Y. P., Guo T., Wang B. J. (2008). Replication of clinical hepatitis B virus isolate and its application for selecting antiviral agents for chronic hepatitis B patients[J]. *World Journal of Gastroenterology*.

[33] Gerner P., Posselt H. G., Krahl A. (2008). Vitamin E treatment for children with chronic hepatitis B: a randomized placebo controlled trial[J]. *World Journal of Gastroenterology*.

[34] Gulcan E. M., Tirit I., Anil A., Adal E., Ozbay G. (2008). Serum neopterin levels in children with hepatitis-B-related chronic liver disease and its relationship to disease severity[J]. *World Journal of Gastroenterology*.

[35] Wang X. L., Xie S. G., Zhang L., Yang W. X., Wang X., Jin H. Z. (2008). Comparison of ligase detection reaction and real-time PCR for detection of low abundant YMDD mutants in patients with chronic hepatitis B[J]. *World Journal of Gastroenterology*.

[36] Lu H.-Y., Zhuang L.-W., Yu Y.-Y. (2008). Effects of antiviral agents and HBV genotypes on intrahepatic covalently closed circular DNA in HBeAg-positive chronic hepatitis B patients[J]. *World Journal of Gastroenterology*.

[37] Lv Y. Y., Shi B. Y., Guo H. (2008). Abrupt onset of type 1 diabetes mellitus during recombinant interferon-alpha 2b therapy in a patient with chronic hepatitis B[J]. *World Journal of Gastroenterology*.

[38] Fan C. L., Wu Y. J., Duan Z. P., Zhang B., Dong P. L., Ding H. G. (2008). Resting energy expenditure and glucose, protein and fat oxidation in severe chronic virus hepatitis B patients[J]. *World Journal of Gastroenterology*.

[39] Zhang Q. I. A. N., Cai D. C., Hu P., Ren H. (2021). Low-level viremia in nucleoside analog-treated chronic hepatitis B patients. *Chinese Medical Journal*.

